RETRACTED

# Study on the Application of the Concept of Childlike Interest with Refined Nursing Intervention in the Treatment of Children with Severe Pneumonia

**DOI:** 10.1155/2022/5360733

**Published:** 2022-08-03

**Authors:** Yuwei Wang, Shuping Qi

**Affiliations:** Department of Pediatrics, Affiliated Zhejiang Hospital, Zhejiang University School of Medicine, China

## Abstract

**Objectives:**

To analyze the application of childlike concept with refined nursing intervention in the treatment of children with severe pneumonia.

**Methods:**

100 cases of children with severe pneumonia admitted to our hospital from June 2019 to June 2021 were selected and divided into the control group and the observation group, in which the control group was given refined nursing care and the observation group was given the childlike concept with refined nursing intervention to compare the treatment effects of patients in both groups. The clinical indexes such as recovery time of body temperature, disappearance time of pulmonary rales, recovery time of heart rate, disappearance time of cough, and hospitalization time, were compared between the two groups.

**Results:**

Compared with the control group, the time to recovery of body temperature, time to disappearance of pulmonary rales, time to recovery of heart rate, time to disappearance of cough, and hospitalization time were significantly lower in the observation group, and the difference was statistically significant (*P* < 0.05). Compared with the control group, the compliance rate of patients in the observation group was significantly lower, and the difference was statistically significant (*P* < 0.05). Compared with the control group, the total effective rate of patients in the observation group was significantly higher, and the difference was statistically significant (*P* < 0.05). Compared with the control group, the overall satisfaction rate of patients in the observation group was significantly higher, and the difference was statistically significant (*P* < 0.05). The results of univariate analysis showed that the differences between the two groups were statistically significant (*P* < 0.05) in terms of economic conditions, payment method, child's condition, child's age, comorbid underlying diseases, and nursing care method, and the results of logistic multifactor regression analysis showed that the payment method of self-payment, child's critical condition, and comorbid underlying diseases were the most important factors affecting the anxiety of the family members of children with severe pneumonia. risk factors for the occurrence of anxiety in the families of children with severe pneumonia, and the method of care was a protective factor (*P* < 0.05).

RETRACTED

**Conclusion:**

The concept of childlike fun and refined nursing interventions can effectively improve the treatment effect of children with severe pneumonia, improve patients' condition, increase patients' compliance and satisfaction, and reduce the risk of anxiety and other negative emotions of the child's family members.

## 1. Introduction

Severe pneumonia refers to a critical stage in the course of pneumonia. Except for the common respiratory symptoms, there are also respiratory failure and other systems obviously involved. The disease is aggravated due to the spread of lung tissue inflammation. Severe pneumonia is a respiratory disease with a high incidence rate all over the world, and it is also a common acute respiratory disease in underage children, mostly caused by bacterial, viral, and other causes with clinical symptoms such as cough, fever, expectoration, and dyspnea [1, 2]. Before the progression of pediatric pneumonia, most of the children have respiratory symptoms. Nonbreastfeeding, malnutrition, air pollution, congenital or acquired immunodeficiency, and premature infants are all high-risk factors for severe pneumonia. The incidence of severe pneumonia in children is high in China. About 21 million children get sick, and about 70000 children died of severe pneumonia every year, which is the primary factor in the death of 5-year-old children [3, 4]. Severe pneumonia often has difficulty in expectoration, causing respiratory failure, heart failure, etc., and seriously endangering the life and health of patients [5]. Refined nursing intervention is grounded on medical science and is in accordance with patients' psychological, physiological, and social needs. Refined nursing emphasizes the “patient-centered” nursing service concept and takes the ultimate goal as improving the physical and mental health of patients. At present, it is widely used in clinical craniocerebral injury and children's nursing. However, due to children's active nature and poor compliance, the treatment effect of children may be affected [6, 7]. Moreover, the children are young and are in the stage of growth and development, which make them have the characteristics of strong susceptibility to disease and low stress ability. Thus, during the treatment process, the discomfort and tolerance caused by the disease are low. Furthermore, the child has poor self-control ability and cannot actively cooperate with nursing operations, which affects the treatment and recovery of the disease. The concept of childlike refers to integrating treatment and nursing into children's emotional cognition through vision, hearing, language, and other means, aimed at improving children's cooperation, alleviating children's pain, and easing the doctor-patient relationship [8]. Refinement nursing makes up for the shortcomings of traditional nursing, emphasizes more on the patient-centered service concept, pays more attention to the actual needs of patients, improves nursing details, advocates active and humanized services, and promotes the entire nursing process to be more comprehensive, systematic, and seamless. In the present study, a total of 100 children with severe pneumonia admitted to our hospital from June 2019 to June 2021 were selected to analyze the application of childlike concept combined with refined nursing intervention in the treatment of children with severe pneumonia.

RETRACTED

## 2. Materials and Methods

### 2.1. General Materials

A total of 100 children with severe pneumonia admitted to our hospital from June 2019 to June 2021 were selected. Inclusion criteria are as follows: (1) The children were treated in PICU of our hospital due to severe pneumonia. (2) The age of children was ≤6 years old. (3) The children's condition was relatively stable and could cooperate with the examination and treatment. The children and their family members were all informed and signed the consent form. Exclusion criteria are as follows: (1) The children with systemic infection. (2) The children with serious functional disorder in important organs. (3) The children with blood system diseases or immune deficiency diseases. (4) The children with nervous system or mental illness. The selected children were randomly divided into the control group and the observation group. There were 50 cases in the control group, including 31 males and 19 females, with an average age of 3.16 ± 1.85 years. There were 50 cases in the observation group, including 28 males and 22 females, with an average age of 3.28 ± 2.04 years. There existed no significant difference in age and sex between the two groups (*P* > 0.05). The selection process of general information is shown in Figure 1.

### 2.2. Methods

The control group was given refined nursing, including strengthening health education, psychological nursing, respiratory nursing, diet nursing, paying close attention to the changes of vital signs of patients before and after discharge, and carrying out effective treatment and intervention.

The observation group was given refined nursing combined with the concept of childlike interest. The concept of childlike interest included visual childlike interest induction, childlike interest cooperation demonstration program, childlike interest simulation experience, and childlike interest game interaction. (1) Choose the wallpaper that children like to decorate the children's ward to create a childlike, quiet, and comfortable environment; place toys that children like in the room to distract children; the ward can be decorated with a variety of light sources to relieve patients' tension, panic, and other negative emotions. (2) Animations such as venipuncture and expectoration can be played in the ward to increase children's sense of bravery. The medical staff should ensure that their actions are gentle and slow during nursing operations to reduce children's tension. (3) Choose a toy that children like as a template to demonstrate various nursing operations with children's attention, so as to increase children's perception of treatment and nursing. Parents can accompany them under certain conditions. (4) Increase the interaction with children, such as asking some childlike questions to distract children's attention and increase their sense of achievement. During the operation, children can be encouraged in a childlike way, and children with good cooperation can be rewarded and praised.

RETRACTED

### 2.3. Outcome Measures

The therapeutic effect is as follows: the therapeutic effect was graded into significant, effective, and invalid. The significant effect was defined as that the symptoms such as cough and pulmonary rales were significantly improved, and the children's vital signs were normal; the effective effect was defined as that the patient's cough, pulmonary rales, and other symptoms were improved, and the children's vital signs tended to be normal; the invalid effect was defined as that the patient's symptoms and vital signs were not improved or even serious.

Clinical indicators are as follows: the changes of vital signs of the patients should be closely observed. The clinical indicators of the two groups should be recorded and compared, such as the recovery time of body temperature, the disappearance time of pulmonary rales, the recovery time of heart rate, the disappearance time of cough, and the hospitalization time.

Compliance is as follows: the self-made compliance analysis scale of our hospital was used, which was divided into complete compliance, partial compliance, and noncompliance. Among them, the children who could fully comply with the nursing operations such as infusion and sputum excretion of medical staff are full compliance; the children could partly comply with the nursing operations such as infusion and sputum excretion of the medical staff, and there was resistance sometimes as part of the compliance; the children's complete failure to cooperate with the nursing operations of the medical staff, such as infusion and expectoration, was regarded as noncompliance.

Satisfaction is as follows: the self-made medical service satisfaction questionnaire of our hospital was used, including quality of life, professional technology, service attitude, and health education. The score range was 0-100 points, of which 90-100 points were very satisfied, 90-80 points were considered as satisfactory, and less than 70 points were considered unsatisfactory. The satisfaction of the two groups was compared.

RETRACTED

### 2.4. Statistical Analysis

The experimental data was analyzed using the SPSS20.0 software. The overall distribution of the measurement data including the age, body temperature recovery time, pulmonary rale disappearance time, heart rate recovery time, cough disappearance time, and the hospitalization time was first checked. The measurement data conforming to the normal distribution were expressed as (*x̅*±*s*), which were determined by the paired sample *t* or two independent samples *t* test. If the data did not conform to the normal distribution, the independent sample rank sum test was used. The enumeration data including the gender, efficacy, satisfaction, and compliance were expressed in % and were compared using the *χ*^2^ text among the different groups; the factors influencing the anxiety of children's family members were analyzed using the logistic multiple regression analysis. *P* < 0.05 is considered statistically significant.

## 3. Results

### 3.1. Comparison of Clinical Symptoms between the Two Groups

Compared with the control group, the observation group had much reduced body temperature recovery time, pulmonary rale disappearance time, heart rate recovery time, cough disappearance time, and the hospitalization time (*P* < 0.05) (Table 1).

### 3.2. Comparison of Compliance between the Two Groups

Compared with the control group, the observation group had significantly higher compliance rate (*P* < 0.05) (Table 2).

### 3.3. Comparison of Curative Efficacy between Two Groups

Compared with the control group, the observation group had obviously higher total effective rate (*P* < 0.05) (Table 3).

### 3.4. Comparison of Patient Satisfaction between the Two Groups

Compared with the control group, the observation group had markedly higher total satisfaction rate (*P* < 0.05) (Table 4).

### 3.5. Univariate Analysis of the Influencing Factors of Anxiety in Family Members of Children with Severe Pneumonia

The results of univariate analysis showed statistically significant differences in terms of economic conditions, payment method, child's condition, child's age, comorbid underlying diseases, and nursing method between the families of children with severe pneumonia with or without anxiety (*P* < 0.05) (Table 5).

RETRACTED

### 3.6. Logistic Multivariate Regression Analysis

The statistically significant factors in Table 5 were taken as independent variables, and whether the family members of children with severe pneumonia had anxiety was taken as dependent variables for logistic multivariate regression analysis. The logistic multifactor regression analysis showed that payment method at own expense, critical illness, and underlying diseases were the risk factors of anxiety in the family members of children with severe pneumonia, and the nursing method was the protective factor (*P* < 0.05) (Table 6).

### 3.7. Nomogram Analysis

Logistic regression analysis results were selected to establish a nomogram of anxiety, and the scores of each predictive index obtained from the nomogram were added to obtain the total score. The corresponding prediction probability was obtained. Different total scores correspond to the probability of anxiety in the family members of children. For example, if a child is paying 90 points for self-pay, 98 points for critical illness, 78 points for combined underlying diseases, 27 points for routine care, and a total score of 293 points, the risk of anxiety is 100% for the patient's family (Figure 2).

### 3.8. ROC Curve Analysis

The results of the ROC curve analysis showed that the areas under the curve of payment at one's own expense, critical illness, underlying diseases, and nursing methods to predict the anxiety of the family members of children with severe pneumonia were 0.674, 0.718, 0.794, and 0.874, respectively (see Table 7 and Figure 3).

## 4. Discussion

Severe pneumonia is a common acute and dangerous lung disease in underage children. The children have higher risk of respiratory tract infection and higher probability of respiratory tract obstruction due to their weak constitution and weaker movement and clearance ability of bronchial cilia than adults. The disease of pneumonia in children is also more serious, which may lead to the death of children [9, 10]. At present, the main treatment for severe pneumonia is anti-inflammatory and improving respiratory symptoms. In severe cases, the respiratory kinetic energy of children can be improved through mechanical ventilation [11]. Some experts also believe that systematic and effective nursing measures have certain significance in improving the treatment effect and prognosis of children [12]. Here, children with severe pneumonia were selected as the research object and the application of childlike interest concept combined with refined nursing intervention in the treatment of children with severe pneumonia was analyzed.

Refined nursing is a nursing concept originated in developed countries. Through the implementation of management, it improves the patience, carefulness, the work quality, and efficiency of medical staff. Refined nursing is widely used in acute and critical diseases such as severe pneumonia and respiratory failure and has good effect [13]. However, due to the immaturity of the child's mental development, severe pneumonia brings physical discomfort and pain to the child, and resistance may occur in the process of treatment and nursing, resulting in poor compliance. Improving the treatment and nursing compliance of children, as well as the treatment effect, have become the focus of medical scholars [14]. The concept of children's interest is a new nursing concept in recent years. It helps children understand the significance of treatment and nursing process through the means of popular science animation and video, question and answer interaction, and the doll demonstration to divert children's attention, improve children's positive and courageous emotions, and increase children's compliance, thereby improving children's treatment effect and recovery speed. At present, child interest management is widely used in retinoblastoma, acute appendicitis, acute lymphoid leukemia, and other diseases. In this present study, the recovery time of body temperature, the disappearance time of pulmonary rales, the recovery time of heart rate, the disappearance time of cough, and the length of hospital stay of the observation group were much reduced than the control group; the total effective rate of patients in the observation group was significantly increased, which was similar to the results of relevant clinical studies [15], suggesting that the concept of child interest combined with refined nursing intervention could effectively improve the treatment effect of children with severe pneumonia and the patient's condition.

RETRACTED

Compared with traditional health education, children's interest management carries out education in a way that children are interested in. It can not only improve children's enthusiasm and initiative but also can increase children's self-confidence and courage, alleviate children's negative emotions such as tension and fear, reduce the incidence of psychological stress events, and reduce medical disputes [16, 17]. In this experiment, the children and their families in the observation group had obviously higher total satisfaction rate and treatment compliance. It can be seen that the concept of child interest combined with refined nursing intervention increase patient compliance and satisfaction and improve the doctor-patient relationship. Logistic regression analysis showed that the concept of childlike interest combined with refined nursing methods was protective factors for the occurrence of anxiety in children's family members. Some scholars have found that systematic and comprehensive nursing intervention given to children and their families on the basis of routine nursing can effectively reduce the anxiety of their families and strengthen the family support system [18]. The results of this study further confirmed the application of the concept of child interest combined with refined nursing intervention in the diagnosis and treatment of patients with severe pneumonia, which solve problems pertinently in the treatment process, strengthen the communication between nurses and children and their families, alleviate the anxiety of children's families, and avoid adverse events affecting the treatment effect.

To sum up, the concept of child interest combined with refined nursing intervention could effectively improve the treatment effect, condition, compliance, and satisfaction of children with severe pneumonia, which could be widely used in clinical practice. However, due to the limited research time and small samples size, the experimental results may be accidental. In our following research, the sample size and research time will be expanded for further exploration.

## Figures and Tables

**Figure 1:** The selection process of general information.

**Figure 2:** Nomogram analysis.

**Figure 3:** ROC curve.

**Table 1:** Comparison of clinical symptoms between the two groups (d, *x̅*±*s*).

Groups	Body temperature recovery time	Pulmonary rale disappearance time	Heart rate recovery time	Cough disappearance time	Hospitalization time
The control group (*n* = 50)	8.56 ± 2.63	6.85 ± 0.85	13.52 ± 3.45	8.16 ± 1.46	14.41 ± 3.15
The observation group (n =50)	6.38 ± 1.89	4.41 ± 1.03	9.71 ± 2.16	5.49 ± 0.98	10.12 ± 1.58
*t*	5.213	14.152	7.250	11.761	9.429
*P*	<0.001	<0.001	<0.001	<0.001	<0.001

**Table 2:** Comparison of compliance between the two groups (cases, %).

Groups	Complete compliance	Partial compliance	Noncompliance	The total compliance
The control group (*n* = 50)	3 (6.00%)	22 (44.00%)	15 (30.00%)	35 (70.00%)
The observation group (*n* = 50)	7 (14.00%)	37 (74.00%)	6 (12.00%)	44 (88.00%)
*χ*^2^				4.882
*P*				0.027

**Table 3:** Comparison of curative efficacy between two groups (cases, %).

Groups	Significant	Effective	Invalid	Total effective
The control group (*n* = 50)	15 (30.00%)	20 (40.00%)	15 (30.00%)	35 (70.00%)
The observation group (*n* = 50)	20 (40.00%)	27 (54.00%)	3 (6.00%)	47 (94.00%)
*χ*^2^				9.756
*P*				0.002

**Table 4:** Comparison of patient satisfaction between the two groups (cases, %).

Groups	Very satisfied	Satisfactory	Unsatisfactory	Total satisfactory
The control group (*n* = 50)	18 (36.00%)	20 (40.00%)	12 (24.00%)	38 (76.00%)
The observation group (*n* = 50)	20 (40.00%)	23 (46.00%)	4 (8.00%)	46 (92.00%)
*χ*^2^				4.761
*P*				0.029

RETRACTED

**Table 5:** Univariate analysis of the influencing factors of anxiety in family members of children with severe pneumonia (cases, %).

Influencing factors		Cases	Anxiety (*n* = 68)	Without anxiety (*n* = 32)	*χ* ^2^	*P*
Gender	Male	59	38 (55.88)	21 (65.63)	0.854	0.355
	Female	41	30 (44.12)	11 (34.38)		
Relationship with the patients	Father	38	27 (39.71)	11 (34.38)	0.263	0.608
	Mother	62	41 (60.29)	21 (65.63)		
Level of education	Primary school	19	14 (20.59)	5 (15.62)		
	Junior and senior high school	34	23 (33.82)	11 (34.38)	0.374	0.829		
	College degree or above	47	31 (45.59)	16 (50.00)		
Economic conditions	≤2000 CNY	24	20 (29.41)	4 (12.50)	7.872	0.020
	2000~5000 CNY	54	38 (55.88)	16 (50.00)		
	>5000 CNY	22	10 (14.71)	12 (37.50)		
Payment method	At one's own expense	56	52 (76.47)	4 (12.50)	36.139	<0.001
	Medical insurance	44	16 (23.53)	28 (87.50)		
Child's condition	Stable	46	18 (26.47)	28 (87.50)	32.628	<0.001
	Critical	54	50 (73.53)	4 (12.50)		
Age	≥3 years	52	25 (36.76)	27 (84.38)	19.761	<0.001
	<3 years	48	43 (63.24)	5 (15.62)		
Comorbid underlying diseases	Yes	54	50 (73.53)	4 (12.50)	32.628	<0.001
	No	46	18 (26.47)	28 (87.50)		
Nursing method	Refined nursing	50	42 (61.76)	8 (25.00)	11.765	0.001
	Childlike interest concept +refined nursing	50	26 (38.24)	24 (75.00)		

**Table 6:** Logistic multivariate regression analysis.

Factors	*B*	*SE*	*Wald*	*P*	OR	95% CI
Economic conditions	0.052	0.182	0.162	0.782	1.052	0.024~1.269
Payment method at own expense	2.147	0.710	9.135	0.001	8.555	2.127~34.416
Critical illness	2.704	0.992	7.429	0.006	4.932	2.137~6.331
Child's age<3 years old	0.415	0.226	0.485	0.135	1.549	0.126~1.987
Comorbid underlying diseases	0.245	0.192	1.244	0.036	1.251	0.048~1.397
Childlike interest concept +refined nursing	-2.318	1.046	4.980	0.013	0.099	0.022~0.758

**Table 7:** ROC curve analysis.

Factors	The areas under the curve	*SE*	*P*	95% CI	Sensitivity (%)	Specificity (%)
Payment at one's own expense	0.674	0.054	<0.001	0.568~0.780	78.00	72.00
Critical illness	0.718	0.051	<0.001	0.619~0.817	80.00	66.00
Comorbid underlying diseases	0.794	0.045	<0.001	0.706~0.881	86.50	72.30
Nursing method	0.874	0.035	<0.001	0.806~0.942	90.20	84.50

## Data Availability

All data generated or analyzed during this study are included in this published article.
